The article "Simultaneous Determination of Gallic Acid, Ellagic Acid, and Eugenol in Syzygium aromaticum and Verification of Chemical Antagonistic Effect by the Combination with Curcuma aromatica Using Regression Analysis" was published in 2013. Journal: J Anal Methods Chem.

# Simultaneous Determination of Gallic Acid, Ellagic Acid, and Eugenol in *Syzygium aromaticum* and Verification of Chemical Antagonistic Effect by the Combination with *Curcuma aromatica* Using Regression Analysis

**DOI:** 10.1155/2013/375294

**Published:** 2013-06-25

**Authors:** Jung-Hoon Kim, Chang-Seob Seo, Seong-Sil Kim, Hyekyung Ha

**Affiliations:** Basic Herbal Medicine Research Group, Korea Institute of Oriental Medicine, Daejeon 305-811, Republic of Korea

## Abstract

This study was designed to perform simultaneous determination of three reference compounds in *Syzygium aromaticum* (SA), gallic acid, ellagic acid, and eugenol, and to investigate the chemical antagonistic effect when combining *Curcuma aromatica *(CA) with SA, based on chromatographic analysis. The values of LODs and LOQs were 0.01–0.11 **μ**g/mL and 0.03–0.36 **μ**g/mL, respectively. The intraday and interday precisions were <3.0 of RSD values, and the recovery was in the range of 92.19–103.24%, with RSD values <3.0%. Repeatability and stability were 0.38–0.73% and 0.49–2.24%, respectively. Compared with the content of reference and relative peaks in SA and SA combined with CA (SAC), the amounts of gallic acid and eugenol were increased, while that of ellagic acid was decreased in SAC (compared with SA), and most of peak areas in SA were reduced in SAC. Regression analysis of the relative peak areas between SA and SAC showed *r* ^2^ values >0.87, indicating a linear relationship between SA and SAC. These results demonstrate that the components contained in CA could affect the extraction of components of SA mainly in a decreasing manner. The antagonistic effect of CA on SA was verified by chemical analysis.

## 1. Introduction

The therapeutic efficacy of herbal formula originates from the combination of two or more herbal medicines and is exerted by the interaction between them. Several types of herbal combinations have been used for the purpose of increasing or enhancing the therapeutic effect, reducing toxicity or the adverse effect, weakening the action of another combined herbal medicine, or causing toxicity or an adverse effect, expressed as “seven types of herbal combination.” Their combinations are expressed as mutual reinforcement, mutual assistance, mutual restraint, mutual suppression, mutual inhibition, and single effect [1]. Besides single effect, mutual reinforcement and mutual assistance have been considered as desirable (and positive) for exhibiting the therapeutic effect (synergistic), while mutual suppression and mutual inhibition have been used due to their aggravating or negative effect (antagonistic). Most reports in the literature have dealt with synergic interactions of herbal medicine such as Astragali radix with Rehmanniae radix to promote diabetic wound healing [2] and *Glycyrrhiza glabra* with *Solanum xanthocarpum* and *Adhatoda vasica* to stabilize mast cells [3]. There are no reports of mutual inhibition or mutual suppression. 

The bud of* Syzygium aromaticum* (SA, syn. *Eugenia caryophyllata*) is a representative herbal medicine of mutual suppression when combined with the radix of *Curcuma aromatica* (CA). SA has been used to treat symptoms such as vomiting, hiccough, abdominal pain, diarrhoea, lack of appetite, vaginal discharge, and weakness of legs for thousands of years in Korea and China. Among its efficacies, reducing vomiting or hiccough and alleviating abdominal pain or diarrhoea are known to be antagonized by the addition of CA [4]. In other words, the therapeutic efficacy of herbal medicine can be reduced or eliminated by combining certain kind of herbal medicine, and hence chemical components of therapeutic efficacy can be also influenced at the levels of the contents or composition.

The pharmacological effects of SA have been reported as antioxidant properties [5], antifungal activity [6], hypoglycaemic effect [7], bone-preserving effect [8], chemopreventive potential for lung cancer [9], regulation of the immune response [10], and antiobesity effect [11]. These effects have mostly been investigated with its extracted essential oil. Owing to the volatile characteristics of its constituents, most of chemical components in SA have been analysed for its essential oil using GC-MS. High concentrations of the volatile compounds such as eugenol, eugenol acetate, *α*- and *β*-caryophyllene, and 1-ethyl-3-nitrobenzene [12–15] were detected. Most quantitative analyses by HPLC have focused on the determination of eugenol [16–18] and other compounds, including gallic acid, ellagic acid, and quercetin glycoside [19]. There is little to be found in the literature on the validated quantitative analysis of those compounds.

In the present study, to evaluate the effect of CA on the constituents of SA, we quantified and then compared the amounts of three reference compounds (gallic acid, ellagic acid, and eugenol) and investigated the variance of the relative peak areas between SA and then SA with CA (SAC) including the three reference compounds. Regression analysis was carried out to determine whether SA and SAC exhibit linear regression and the influence of the addition of CA to SA. 

## 2. Materials and Methods

### 2.1. Reagents and Plant Materials

Methanol, acetonitrile, and water (HPLC grade) were purchased from JT Baker Inc. (Phillipsburg, NJ, USA). Gallic acid, ellagic acid, and eugenol were purchased from Sigma-Aldrich (St Louis, MO, USA). The purity of all standard compounds was >98% except for ellagic acid (95%). The chemical structures of the standard compounds are shown in Figure 1. The herbal medicines were purchased from the herbal medicine company Kwangmyungdang Medicinal Herbs (Ulsan, Korea). A voucher specimen (2012-EBM88-90) has been deposited in the Basic Herbal Medicine Research Group of the Korea Institute of Oriental Medicine.

### 2.2. Preparation of Sample Extract

A 100 g quantity of dried powder of each sample (SA, CA and SAC) was extracted by 2 h reflux with 1000 mL distilled water at 100°C. An extract was centrifuged at 3000 rpm for 10 min and the supernatant filtered through a paper filter, and then it was lyophilized to create a powder. Accurately weighed SA, CA and SAC samples (20 mg) were dissolved separately in 20 mL distilled water and filtered through a 0.2 *μ*m syringe filter (SmartPor, Woongki Science, Seoul, Korea) prior to the HPLC injections. 

### 2.3. Preparation of Standard Solutions

The standard compounds were accurately weighed and then dissolved in methanol to prepare stock solutions in concentrations of 1000 *μ*g/mL. The stock solutions containing the standard compounds were diluted to produce working solutions, which were used to construct calibration curves.

### 2.4. Chromatographic Instrumentation and Conditions

The HPLC system comprised a Shimadzu LC-20A (Kyoto, Japan) equipped with a solvent delivery unit (LC-20AT), autosampler (SIL-20AC), column oven (CTO-20A), degasser (DGU-20A_3_), and photodiode array detector (SPD-M20A). The acquired data were processed using LabSolutions software (Ver. 5.3; Shimadzu, Japan). Separation was performed on a Gemini C_18_ column (4.6 × 250 mm, 5 *μ*m; Phenomenex, Torrance, CA, USA) maintained at 40°C. The mobile phase consisted of water (A) and acetonitrile (B), both containing 1% acetic acid. Gradient elution of the mobile phase was applied: 5–70% (B) over 0–30 min, 70–100% (B) over 30–35 min, held for 5 min. The flow rate was 1.0 mL/min and the injection volume was set to 10 *μ*L. The detection wavelengths were optimized according to the maximum absorption wavelengths of standard compounds: gallic acid at 280 nm, ellagic acid at 254 nm, and eugenol at 280 nm.

### 2.5. Method Validation

The within-day (intraday) and between-day (interday) precisions were calculated by analysing sample extracts added by three different concentration levels of reference compounds (low, medium, and high) with values determined as RSD. The accuracy of the method used was investigated by means of a recovery test, which involved adding three different concentration levels of reference compounds (low, medium, and high) to the samples, followed by extraction using the methods described above. The recovery was calculated as follows: recovery (%) = ((detected concentration − original concentration)/spiked concentration) × 100. The repeatability was evaluated by five replicates of SA solutions and the stability was determined by SA solution prepared over five consecutive days. Both values were expressed as RSD values.

### 2.6. Statistical Analysis

All experiments were performed at least three times. The peaks that showed differences between SA and SAC were chosen and their relative areas to total area were calculated. Student's paired *t*-test was used to test whether the mean of each peak differed significantly. Regression analysis on the peaks that influenced the difference between samples was performed using open-source software “R (ver. 2.15.1)”.

## 3. Results and Discussion

### 3.1. Linear Regression, LOD and LOQ

Stock solution containing the reference compounds was diluted to eight levels of concentration to construct calibration curves. The correlation coefficient (*r* ^2^) of compounds ranged from 0.9996 to 0.9998, showing good linearity. The values of LODs and LOQs calculated by the concentrations of each compound at signal-to-noise ratios of 3 and 10 were as follows: LOD = 0.01–0.11 *μ*g/mL and LOQ = 0.03–0.36 *μ*g/mL (Table 1). All the reference compounds were well detected and separated on chromatograms at their maximum absorption wavelengths using the methods described in Figure 2(a).

### 3.2. Method Validation

The precisions of the reference compounds were represented as RSD values, calculated as the percentage of standard deviation divided by the mean value. The RSD values of the intra-day and inter-day precisions ranged from 0.12% to 2.57% and 0.08% to 2.26%, both being <3.0 (Table 2). The recoveries of the reference compounds were in the range 92.19–103.24%, with RSD values <3.0% (Table 3). Repeatability and stability of each compound ranged from 0.38% to 0.73% and 0.49% to 2.24%, respectively (Table 4). 

### 3.3. Determination of the Reference Compounds in Samples

As shown in Figure 3, noticeable variances were observed in the content of the three reference compounds, which exhibited predominant peak height and area in the chromatograms. Eugenol, the major constituent of SA, was responsible for most of the pharmaceutical effects, such as anti-giardiasis [20], inhibition of B16 melanoma cells [21], gastroprotective activity [22]. Gallic acid and ellagic acid, although not predominant in SA, reported to have pharmacological effects such as anticancer activity [23, 24] and cardioprotective [25], antiatherogenic [26], and anti-inflammatory effects [27]. The three compounds, being abundant in the extract, are thought to contribute to the therapeutic effect of SA. 

There was a slightly higher content of gallic acid in the SAC extract (18.51 ± 0.26 mg/g) than in the SA extract (17.76 ± 0.08 mg/g). The content of ellagic acid in the SA extract (16.27 ± 0.03 mg/g) was decreased about 0.4-fold in the SAC extract (6.70 ± 0.08 mg/g), whereas that of eugenol in the SA extract (37.65 ± 0.20 mg/g) was rather increased about 1.6-fold in the SAC extract (59.00 ± 0.02 mg/g). These results indicate that the extraction rates of the three reference compounds in the SA extract might be influenced by the combination of CA, which means that some unknown components in CA could affect the extraction efficiency of gallic acid, ellagic acid, and eugenol in SA extract. A change in amounts of predominant compounds in SA might weaken or strengthen the therapeutic effect of SAC. 

### 3.4. Investigation of the Influence of CA on SA

As shown Figure 2, overall chromatogram patterns of SA and SAC are similar after a retention time of 5 min. In contrast, the chromatogram of CA did not show any noteworthy peaks, except at a retention time <5 min. To investigate the degree of influence of CA on SA, the peaks that showed the same retention time between SA and SAC were selected and their relative areas to total peak area were calculated. Overall, 21 peaks (including gallic acid, ellagic acid, and eugenol) were selected excluding the peaks that eluted at <5 min (Figures 2(b) and 2(c)). The relative area ratio of each selected peak was calculated using the areas of peaks in SA extract divided by those in SAC extract. A ratio of 1.0 means there was no change in peak area between SA and SAC; a ratio of <1 or >1 means the peak areas detected in SAC extract were affected by the combination of CA and SA. The ratios of gallic acid, eugenol, and peak 3 were >1.0, whereas those of 18 peaks (including ellagic acid) were <1.0, even <0.1 at peak 1 and peak 7 (Figure 4). We believe that the combination of CA can affect the extraction of constituents in SA by decreasing the content of most components or increasing that of several components, which means the components in CA might interrupt or accelerate the extraction of components in SA according to their interaction.

These results were confirmed by regression analysis of the relative area of peaks between SA and SAC. We set the relative peak areas in SA as independent variables and those in SAC as dependent variables. The peaks were distributed close to the equation line, except those of gallic acid, ellagic acid, and eugenol, which were considered as outliers (Figure 5). The slope of the linear equation was 1.020356 with a *P* value < 0.001, the correlation coefficient (adjusted *r* ^2^) was 0.8879, and the *F*-statistic was 135.7 with a *P*-value < 0.001, which means that dependent variables (SA) are casually related to independent variables (SAC). A similar interpretation is reported in the literature [28] (Table 5). Our results further confirm that adding CA to SA affects the extraction efficiency of the components from SA, which is supported by regression analysis because SAC (consisting of two herbal medicines, SA and CA) have a linear relation with SA; hence, CA is only a contribution in verifying the variance of components in SA. 

To assess the linear regression, we performed the assumption of homogeneity of variance and normality by examining the residuals.  Figure 6 shows the trend in the model residuals; there was decreasing variance from left to right but the trend line was increased to the region of gallic acid, ellagic acid, and eugenol far from the mainly distributed region (e.g., Figure 6(a)). In the normal Q-Q (quantile-quantile) plot, residual errors were normally distributed along the line except for gallic acid, ellagic acid, and eugenol away from the centre (e.g., Figure 6(b)). Similar to the “residauls versus fitted plot,” the “scale-location plot” also showed the trend line through the mean of the plots and the line elongates to the three reference compounds (e.g., Figure 6(c)). In the “residuals versus leverage” plot, the densely gathered points were on the left side of the horizontal line with leverage <0.1 with the trend line passing the centre of the cluster. However, the three reference compounds (gallic acid, ellagic acid and eugenol) were located at high leverage >0.2, and Cook's distance was close to 0.5 for gallic acid and >1 for ellagic acid, and eugenol, which means that these compounds could be considered as outliers (e.g., Figure 6(d)). 

When putting those four plots together, we observed little normality and the three reference compounds (gallic acid, ellagic acid, and eugenol) were determined as possible outliers responsible for violating the constant variance. However as gallic acid, ellagic acid, and eugenol were evaluated as the most influential factors in the regression model and were abundant in samples, excluding them does not benefit to investigate the effects of adding CA on the extraction efficiency of the component in SA. 

## 4. Conclusions

The components in SA could be influenced by the combination thereof with CA, with most showing decreasing trends in their amounts, indicating that the components in CA can interfere with the extraction of components from SA. We verified the antagonistic effect of CA on SA by quantitative determination and regression analysis by means of chemical analysis. These results would be definitive with further supportive biological assay. 

## Figures and Tables

**Figure 1:** Chemical structures of three standard compounds in *Syzygium aromaticum* extract: (**1**) gallic acid, (**2**) ellagic acid, and (**3**) eugenol.

**Figure 2:** HPLC chromatograms of water extracts of *Syzygium aromaticum *(SA, A), *Syzygium aromaticum *combined with* Curcuma aromatica* (SAC, B), and *Curcuma aromatica* (CA, C) at the detection wavelength of 280 nm. Peaks 1–18: unidentified compounds: (a) Overall chromatogram within 30 min, (b) segmented chromatogram from 2.5 min to 15 min, and (c) segmented chromatogram from 15 min to 30 min.

**Figure 3:** Comparison of the contents of gallic acid, ellagic acid, and eugenol in *Syzygium aromaticum *(SA) and *Syzygium aromaticum *combined with* Curcuma aromatica* (SAC). Significance of difference represented as **P < 0.01 and ***P < 0.001.

**Figure 4:** Relative area ratio of the 18 selected peaks in the chromatogram of *Syzygium aromaticum *(SA) and *Syzygium aromaticum *combined with* Curcuma aromatica* (SAC). The ratios mean relative peak areas of SAC divided by those of SA.

**Figure 5:** Linear regression plot of relative peak areas between *Syzygium aromaticum *(SA) and *Syzygium aromaticum *combined with* Curcuma aromatica* (SAC) except for outliers (gallic acid, ellagic acid, and eugenol). Peak 1–18: unidentified compounds.

**Figure 6:** Assessment of regression analysis with residuals between relative peak areas of *Syzygium aromaticum *(SA) and *Syzygium aromaticum *combined with* Curcuma aromatica* (SAC). Dot numbers of 2, 13 and 21 represent gallic acid, ellagic acid, and eugenol, respectively.

**Table 1:** Linear regression, correlation coefficients (*r* ^2^), LOD, and LOQ for the reference compounds (*n* = 3).

Compound	Linear equation	Correlation coefficient	Linear range (*μ*g/mL)	LOD^a^ (*μ*g/mL)	LOQ^b^ (*μ*g/mL)
Gallic acid	*y* = 32700.38*x* − 18582.04	0.9998	0.78–100	0.05	0.16
Ellagic acid	*y* = 88471.48*x* − 48062.58	0.9998	0.78–100	0.01	0.03
Eugenol	*y* = 10497.31*x* − 8692.62	0.9996	1.56–200	0.11	0.36

^a^Limit of detection, ^b^limit of quantification.

**Table 2:** Intraday and interday precision of three reference compounds in *Syzygium aromaticum* extract (*n* = 3).

Compound	Spiked concentration (*μ*g/mL)	Intraday		Interday	
		Detected concentration (*μ*g/mL)	RSD^a^ (%)	Detected concentration (*μ*g/mL)	RSD (%)
Gallic acid	5	5.03	2.57	5.30	1.77
	10	9.64	1.80	9.59	2.02
	20	20.17	0.42	20.13	0.58

Ellagic acid	5	5.34	0.78	5.45	2.80
	10	9.67	2.14	9.88	2.26
	15	15.11	0.95	14.93	1.27

Eugenol	10	10.52	0.83	10.39	0.36
	25	25.09	0.28	25.16	0.14
	40	39.81	0.12	39.81	0.08

^a^Relative standard deviation (%) = (standard deviation/mean) × 100.

**Table 3:** Recovery of 3 reference compounds in the *Syzygium aromaticum* extract (*n* = 6).

Compound	Original concentration (*μ*g/mL)	Spiked concentration (*μ*g/mL)	Detected concentration (*μ*g/mL)	Recovery (%)	RSD^a^ (%)
Gallic acid	17.76	5	22.80	102.16	2.56
		10	27.39	96.37	1.44
		20	37.99	101.03	0.97

Ellagic acid	16.27	5	21.41	102.81	0.13
		10	25.49	92.19	1.66
		15	30.61	95.62	2.36

Eugenol	37.72	10	48.08	103.24	0.64
		25	62.24	97.98	0.33
		40	76.34	96.51	0.11

^a^Relative standard deviation (%) = (standard deviation/mean) × 100.

**Table 4:** Repeatability and stability of three reference compounds in *Syzygium aromaticum* extract (*n* = 5).

Compound	Repeatability (RSD, %)	Stability (RSD, %)
Gallic acid	0.73	0.70
Ellagic acid	0.38	2.24
Eugenol	0.66	0.49

**Table 5:** Regression analysis of the relative peak areas between *Syzygium aromaticum *(SA) and *Syzygium aromaticum *combined with* Curcuma aromatica* (SAC).

Coefficients	*R*-squared	*F*-statistic	*P*-value
Slope 1.211039 Pr(>|*t*|) 3.83 × 10^−10^	0.8722	137.5	3.835 × 10^−10^
